# *Citrus unshiu* Peel Attenuates Dextran Sulfate Sodium-Induced Ulcerative Colitis in Mice due to Modulation of the PI3K/Akt Signaling Pathway and MAPK and NF-*κ*B

**DOI:** 10.1155/2022/4041402

**Published:** 2022-05-17

**Authors:** Se Hui Lee, Jin A. Lee, Mi-Rae Shin, Hae-Jin Park, Seong-Soo Roh

**Affiliations:** ^1^Department of Herbology, College of Korean Medicine, Daegu Haany University, Daegu 42158, Republic of Korea; ^2^DHU Bio Convergence Testing Center, Daegu Haany University, 1, Hanuidae-ro, Gyeongsan-si 38609, Republic of Korea

## Abstract

**Aim:**

*Citrus unshiu* peel has been used to treat various diseases in traditional East Asian medicine including Korea, and many studies have been reported regarding inflammatory diseases including ulcerative colitis (UC). However, the underlying mechanism by which *Citrus unshiu* peel modulates inflammation in UC remains unclear. Therefore, this study aimed to evaluate the therapeutic effect and underlying mechanism of *Citrus unshiu* peel water extract (CUP) for UC.

**Methods:**

The experiment for UC was conducted with 8-week-old male Balb/c mice. After 1 week of adaptation, acute colitis was induced in all groups except the normal group by 5% DSS dissolved in drinking water for 1 week. Balb/c mice were divided into 5 groups (*n* = 8/group): control group (Control), distilled water-treated group (DSS), 100 mg/kg sulfasalazine-treated group (SASP), 100 mg/kg CUP-treated group (CUPL), and 200 mg/kg CUP-treated group (CUPH). The efficacy of CUP on UC was evaluated by biochemical analyses such as ROS and MPO in serum and MDA in tissues, and expression of proteins related to inflammation and apoptosis was evaluated through Western blot.

**Results:**

As a result of confirming the macroscopic changes and H&E staining in colon tissues to confirm the preventive and therapeutic effects of CU, decrease in colon length and inflammatory lesions were inhibited in the CUP-treated group compared to the DSS group. In addition, as a result of serum ROS and tissue MDA analysis and oxidative stress-related protein analysis, it was significantly decreased in the CUP-administered group compared to the control group. In addition, treatment with CUP not only inactivated MAPK, p-I*κ*B*α*, and NF-*κ*Bp65 by blocking the PI3K/Akt pathway but also significantly reduced the expression of inflammatory cytokines.

**Conclusion:**

These results show that CUP not only suppresses oxidative stress in UC but also regulates inflammation-related proteins and apoptotic proteins by regulating the PI3K/Akt signaling pathway, suggesting that it has the potential as a material for developing new natural therapeutic agents for UC.

## 1. Introduction

Inflammatory bowel disease (IBD) is increasing in developed as well as developing countries, and it is receiving considerable attention as a global public health problem [1, 2]. In addition, according to a study recently published in the journal *Lancet Gastroenterol Hepatol*, there were 6.8 million cases of IBD in 2017 [3]. IBD, a chronic and recurrent inflammatory disease, repeatedly exhibits inflammatory responses due to various causes in the small and large intestine and is largely divided into ulcerative colitis (UC) and Crohn's disease (CD) [4]. Herein, UC is a gastrointestinal disorder characterized by inflammatory lesions of the rectal and colonic mucosa. Clinical symptoms include diarrhea, bloody stools, abdominal pain, mucus, and pus, which cause repeated seizures, seriously affecting the physical and mental health of the patient [5]. Although the specific etiology of UC is not yet clear, the pathogenesis of these diseases may be associated with inflammation, genetic factors, epithelial barrier defects, infections, and immune disorders [6]. So far, the medical treatment of IBD including UC and CD has only been palliative therapies, such as anti-inflammatory drugs, immunosuppressants, and corticosteroids [7, 8]. Unfortunately, these treatments are only adjuvant, with limited efficacy and serious side effects when taken over long periods of time. Therefore, there is an urgent need to develop a therapeutic agent that has fewer side effects and is excellent for treating inflammation, and it is urgent to elucidate the exact etiology.

*Citrus unshiu* peel (*Citrus reticulata*) is the bark of *Citrus unshiu* Markovich and has been widely used for the treatment of blood circulation disorders, asthma, indigestion, and vomiting in East Asia including Korea, Japan, and China since ancient times [9]. Components isolated from *Citrus unshiu* peel include narirutin, hesperidin, and *β*-carotene [10]. Also, in a recent study, *Citrus unshiu* peel was shown to have various pharmacological effects against viral infection, depression, obesity, and inflammation [11–14]. In the studies of Noh et al. and Karthikeyan et al., it was reported that the *Citrus unshiu* peel exhibits anti-inflammatory effects in LPS stimulated RAW264.7 [15, 16], and in the study of Nishi et al., the *Citrus unshiu* peel relieves inflammation through the NF-*κ*Bp65 and MAPK pathways in the model of systemic inflammation [17].

Therefore, based on these previous studies, the purpose of this study was to elucidate the therapeutic effect and mechanism of action of *Citrus unshiu* peel water extract (CUP) in a mouse model of 5% DSS-induced UC.

## 2. Materials and Methods

### 2.1. Materials

Dextran sodium sulfate (DSS) was purchased from MP Biologicals (Santa Ana, CA, USA). Aluminium chloride was purchased from Thermo Fisher Scientific (Ward Hill, MA, USA). Potassium persulfate, sulfasalazine (purity ≥98%), dithiothreitol (DTT), potassium phosphate monobasic, potassium phosphate dibasic, sodium hydroxide, 1,1,3,3-tetramethoxypropane, phenylmethanesulfonyl fluoride (PMSF), and 2-thiobarbituric acid (TBARS) were purchased from Sigma-Aldrich (St Louis, MO, USA). 2′,7′ Dichlorofluorescein diacetate (DCFH-DA) was purchased from Molecular Probes (Eugene, OR, USA). Potassium acetate and sodium carbonate were purchased from Daejung Chemicals & Metals Co., Ltd. (Siheung, Korea). Phosphoric acid was purchased from Duksan Company (Ansan, Korea). The protease inhibitor mixture solution and ethylene diamine tetraacetic acid (EDTA) were purchased from Wako Pure Chemical Industries, Ltd. (Osaka, Japan). The required pierce bicinchoninic acid (BCA) Protein Assay Kit for protein quantification was purchased from Thermo Fisher Scientific (Waltham, MA, USA). ECL Western Blotting Detection Reagents and pure nitrocellulose membranes were purchased from GE Healthcare (Chicago, IL, USA) and used. Mouse polyclonal antibodies against NOX2 (SC-7271), p47^phox^ (SC-17845), p22^phox^ (SC-271968), PI3K (SC-1637), p-p38 MAPK (SC-7973), p-ERK (SC-7383), p-JNK (SC-6254), c-Fos (SC-166940), NF-*κ*Bp65 (SC-8008), I*κ*B*α* (SC-1643), p-I*κ*B*α* (SC-8404), iNOS (SC-7271), Cox-2 (SC-19999), Bax (SC-7480), Bcl-2 (SC-7382), caspase-3 (SC-56053), survivin (SC-17779), histone (SC-8030), and *β*-actin (SC-47778), rabbit polyclonal antibodies against ERK 1/2 (SC-292838) and JNK (SC-571), and goat polyclonal antibodies against TNF-*α* (SC-1351), IL-6 (SC-1266), and IL-1*β* (SC-1252) were purchased from Santa Cruz Biotechnology, Inc. (Dallas, TX, USA). Rabbit polyclonal antibodies against p-PI3K (#4228), Akt (1 : 1,000, #9272), p-Akt (#9275), and p38 MAPK (#9212) and mouse polyclonal antibodies against c-Jun (1 : 1,000, #2315) were purchased from Cell Signaling Technology, Inc. (Danvers, MN, USA). And, goat anti-mouse (GTX213111-01), rabbit anti-goat (GTX228416-01), and goat anti-rabbit (GTX213110-01) immunoglobulin G (IgG) horseradish peroxidase (HRP)-conjugated secondary antibodies were purchased from GeneTex, Inc. (Irvine, CA, USA).

### 2.2. Preparation of the Plant Material

*Citrus unshiu* peel was supplied from Bonchowon (Yeongcheon-si, Gyeongsangnam-do) and used. 10 times water was added to 300 g of dried *Citrus unshiu* peel from herbs and extracted at 100°C for 2 hours using a hot water extractor (Daewoong Bio, DWT-1800T, Hwaseong, Korea). After filtration, the extraction solvent was evaporated at 50°C using a rotary evaporator (Buchi B-480, Buchi Labortechnik AG, Flawil, Switzerland). Then, the solvent was evaporated *in vacuo* using a freeze dryer (LABCONCO, Kansas, MO, USA) to obtain the extract in a yield of 9.3%, and *Citrus unshiu* peel water extract (CUP) powder was stored at −80°C.

### 2.3. Analysis of Narirutin and Hesperidin

The water extract of *Citrus unshiu* peel (0.5 mg) was dissolved in 1 mL of 100% methanol and centrifuged at 13,500 rpm for 3 minutes, and the supernatant was analyzed. The solution was injected (1 *μ*L) into a Waters Acquity UPLC system (Waters®, Milford, MA, USA) with a reversed-phase C18 column (Phenomenex 2.6 *µ*m C18 100 Å, 2.1 × 100 mm, Phenomenex, Torrance, CA, USA). The solvent system used was as follows: solvent A (deionized water with 0.1% formic acid), solvent B (100% acetonitrile with 0.1% formic acid); A:B = 82 : 18 -> 82 : 18 (1 min) -> 75 : 25 (15 min) -> 0 : 100 (20 min) -> 0 : 100 (25 min) -> 82 : 18 (26 min) -> 82 : 18 (32 min) at a flow rate of 0.2 mL/min with a UV absorption monitoring (284 nm). The peaks of narirutin and hesperidin were assigned by comparison of retention times (hesperidin: 9.964 min, narirutin: 7.983 min) and UV spectra of authentic standards. Quantification of narirutin and hesperidin in the extract was performed by peak area measurement. The peak areas of 0.3125, 0.625, 1.25, 2.5, 5, 10, 20, and 40 *μ*g/mL were repeated 5 times to create a calibration curve for the genuine standard. The regression coefficients (R2) of the narirutin and hesperidin calibration curves were calculated to be 0.9999 and 0.9992, respectively.

### 2.4. Induction of Ulcerative Colitis and Treatment

These animal experiments protocols were performed according to the “Guidelines for Animal Testing” approved by the Ethics Committee of Daegu Haany University (ulcerative colitis induced with DSS in mice; Approval No. DHU2021-093). The 8-week-old male Balb/c mice (20–24 g) were purchased from DBL (Eumseong, Korea) and used for experiments. After 1 week of adaptation in an animal room controlled by temperature (22 ± 2°C), humidity (50% ± 5%), and a 12-hour light-dark cycle, a total of 40 mice were randomly grouped into 5 groups as follows:

We followed the methods of Shin et al. [18] and Mathew et al. [19].

1. Control group, received D.W. only.
2. DSS group, 5% DSS-induced UC treated with D.W.
3. SASP group, 5% DSS-induced UC treated with sulfasalazine (100 mg/kg).
4. CUPL group, 5% DSS-induced UC treated with CUP (100 mg/kg).
5. CUPH group, 5% DSS-induced UC treated with CUP (200 mg/kg).

All mice except the control group were given 5% DSS dissolved in distilled water for 7 days. At the same time, the drug was orally administered to each group, and the body weight and the amount of water were measured at a fixed time. On the 7th day, only drinks were served after an 18-hour fast. On the 8th day, inhalation anesthesia was performed with isoflurane (Troikaa Pharmaceuticals Ltd, Gujarat, India), and the blood collected from the heart was centrifuged using a centrifuge (GYROZEN Co. Ltd., LaboGene 1730R, Gimpo, Korea). The serum and colon tissue were stored frozen (−80°C).

### 2.5. Measurement of Glutamic Oxaloacetic Transaminase (GOT) and Glutamate Pyruvate Transaminase (GPT) Levels

Liver function parameters such as GOT and GPT in serum were measured using an assay kit (Asanpharm Co., Ltd, Seoul, Korea).

### 2.6. Measurement of Myeloperoxidase (MPO) Levels

MPO was measured using serum, and the level was measured according to the protocol of the MPO colorimetric activity assay kit (BioVision, CA, USA).

### 2.7. Measurement of Reactive Oxygen Species (ROS) in Serum and Malondialdehyde (MDA) in Tissue Levels

ROS level was measured referring to the method of Ali et al. [20]. After mixing well with serum and 1 mM EDTA-50 mM sodium phosphate buffer (pH 7.4), 0.125 mM DCFH-DA was added, then the emission of 535 nm and change of fluorescence values at 485 nm excitation were confirmed. And the absorbance of each well was measured for 30 min at 5-min intervals using a UV-VIS spectrophotometer (Infinite F200 pro, Tecan, Switzerland). MDA level was measured by the method [21]. After mixing the 1% phosphoric acid and sample, 0.67% thiobarbituric acid was added and heated (95°C for 45 min). Then, butanol was mixed and centrifuged (3,000 rpm for 10 min), and the absorbance value of the supernatant was measured using a microplate reader (540 nm). And 1,1,3,3,-tetramethoxypropane was used as a standard material in this experiment.

### 2.8. Preparation of Nuclear and Cytosol Factions and Western Blotting

For cytosol samples, colon tissues were lysed with buffer A containing 0.1 mM phenylmethyl sulfonyl fluoride, 0.1 mM EDTA, 10 mM KCl, 1 mM DTT, 10 mM HEPES (pH 7.8), 2 mM MgCl_2_, and 1,250 *μ*L protease inhibitor solution (Wako). Colon tissues were homogenized using a Homogenizer Stirrer (DAIHAN Scientific Co., Ltd., HS-30E, Wonju, Korea), and the homogenate was incubated for 30 minutes. Then, mixed with 10% NP-40 and centrifuged (12,000 rpm for 2 min at 4°C), the supernatant was collected as a cytosol sample. After that, wash twice with buffer A (washing buffer) with NP-40 (10%) added, and 100 *μ*L of buffer C (10% glycerol, 50 mM KCl, 0.3 mM NaCl, 0.1 mM PMSF, 50 mM HEPES, and 0.1 mM EDTA) was added and resuspended, followed by vortexing three times at 10-minute intervals. Samples were centrifuged at 12,000 rpm at 4°C for 10 min, and the supernatant collected was the nuclear sample. Then, centrifugation (12,000 rpm, 4°C, 10 min) was performed to obtain a supernatant containing the nuclear, and the cytosol and nuclear were stored frozen (–80°C), respectively. Samples containing 10 *μ*g of protein were electrophoresed through 8–14% SDS-PAGE and transferred to a nitrocellulose membrane (GE Healthcare, Chicago, IL, USA). After attaching the primary antibody (1 : 1000) and secondary antibody (1 : 3000) to be analyzed to each membrane, it was visualized using an ECL reagent. Each band was detected by Sensi-Q 2000 Chemidoc (Lugen Sci Co., Ltd., Gyeonggi-do, Korea). We followed the methods of Shin et al. [18].

### 2.9. Statistical Analysis

The data were expressed as means ± SD. Statistical comparisons were analyzed by one-way ANOVA tests using SPSS (version 26.0, IBM, Armonk, NY, USA); after that, posttest statistical significance was determined using the least significant difference (LSD) test. Values of *p* < 0.05, *p* < 0.01, and *p* < 0.001 were considered significant.

## 3. Results

### 3.1. *Citrus unshiu* Peel Analysis by HPLC Chromatogram

Flavonoids belonging to phenolic compounds, which are polyphenols of plants, show various effects such as antibacterial, anti-inflammatory, anticancer, and antioxidant actions and are known to reduce natural antioxidants and inflammatory markers [22]. Hesperidin and narirutin are known as citrus flavonoids, and studies on antioxidant and anti-inflammatory properties using hesperidin, narirutin, and *Citrus unshiu* peel extract, which are components isolated from the *Citrus unshiu* peel, are being actively conducted [23, 24]. The amounts of narirutin and hesperidin in the water extract of *Citrus unshiu* peel were analyzed to be 12.210 ± 0.311 and 9.998 ± 0.146 (mg/g, mean ± SEM), respectively (Figure 1).

### 3.2. Effect of CUP on Changes in Body Weight, Colonic Tissue Length, Biochemical Analysis, and Histological Analysis

As shown in Figures 2(a) and 2(b), we first measured the effects of sulfasalazine and CUP on weight change and reduction in colon length. Compared with the control group, the DSS group had a significant decrease in body weight (*p* < 0.001), but compared to the DSS group, the SASP group and the CUP-treated group significantly inhibited the weight loss. In addition, compared to the control group, the DSS group showed a significant decrease in colon length (*p* < 0.001), but compared to the DSS group, the SASP group and the CUP treatment group showed a tendency to suppress, although not significantly, the decrease in colon length. As can be seen in Figure 2(c), the level of MPO was increased 1.64-fold in the DSS group compared to the control group (*p* < 0.01), whereas the SASP group and the CUPH group significantly decreased 30% (*p* < 0.01), and the CUPL group also significantly decreased 23% (*p* < 0.05). In addition, the results of analyzing the histological changes in the colon tissue are shown in Figure 2(d). The loss of colonic muscle fragments and inflammatory cell infiltration were observed in the DSS group compared to the control group. Inflammatory lesions including loss of colonic muscle fragment and inflammatory cell infiltration were decreased in SASP and CUP treatment groups compared to the DSS group. In addition, these histological changes were quantified by the infiltration of inflammatory cells using the ImageJ program. The value was significantly increased in the DSS group (*p* < 0.001) compared to the control group and was significantly decreased in the SASP group (*p* < 0.001) and the CUP-treated group (*p* < 0.001) compared to the DSS group (Figure 2(e)).

### 3.3. CUP Improved Liver Function Indicator Analysis GOT and GPT in Serum

In order to indirectly confirm drug-induced liver damage, GOT and GPT, which are liver function index analyzes, were measured. As can be seen in Figures 3(a) and 3(b), the level of GOT increased 2.22-fold in the DSS group compared to the control group (*p* < 0.001), whereas it was significantly decreased compared to the DSS group in the SASP group and the CUP-treated group (SASP, 48%, *p* < 0.001; CUPH, 39%, *p* < 0.001, respectively). The level of GPT was increased 1.1-fold in the DSS group compared to the control group (*p* < 0.01), whereas there was a significant decrease by 12% in the SASP group (*p* < 0.01) and a significant decrease by about 7% in the CUPL and CUPH groups (*p* < 0.05).

### 3.4. CUP Suppressed Oxidative Stress Biomarkers and NADPH-Related Proteins

Oxidative stress biomarkers including serum ROS and tissue MDA were evaluated (Figures 4(a) and 4(b)), and the levels of NOX2 and p47^phox^ were evaluated through Western blotting (Figure 4(c)). Serum ROS and tissue MDA levels were significantly increased in the DSS group compared to the control group (ROS level, 1.6-fold, *p* < 0.001; MDA level, 1.4-fold, *p* < 0.001, respectively), whereas in the SASP group and CUPH group, the ROS level was significantly decreased by about 15% (*p* < 0.01, respectively) and the MDA level was significantly decreased by about 25% (*p* < 0.01, respectively). The expression levels of NOX2 and p47^phox^ in the DSS group were significantly higher than those in the control group and increased 1.45- and 1.30-fold, respectively. In the SASP and CUPH group, the levels of NOX2 and p47^phox^ decreased significantly (SASP, 29%, *p* < 0.01; 25%, *p* < 0.001; CUPH, 18%, *p* < 0.01; 18%, *p* < 0.01, respectively).

### 3.5. CUP Activated the PI3K/Akt Signaling

The levels of p-PI3K and p-Akt were evaluated through Western blotting (Figure 5). Compared with the control group, p-PI3K and p-Akt were significantly increased in the DSS group (1.60-fold, *p* < 0.001; 1.35-fold, *p* < 0.001, respectively), and compared to the DSS group, the SASP group (p-PI3K, 30%, *p* < 0.001; p-Akt, 21%, *p* < 0.001, respectively) and CUPH group (p-PI3K, 27%, *p* < 0.001; p-Akt, 26%, *p* < 0.001, respectively) were significantly decreased.

### 3.6. CUP Suppressed c-Fos, c-Jun, and MAPK Proteins in DSS-Induced Colon Tissue

The levels of c-Fos, c-Jun, and MAPK proteins were evaluated through Western blotting (Figure 6). Compared with the control group, c-Fos and c-Jun were significantly increased in the DSS group (1.68-fold, *p* < 0.001; 1.61-fold, *p* < 0.001, respectively), and compared to the DSS group, the SASP group (c-Fos, 21%, *p* < 0.001; c-Jun, 26%, *p* < 0.001, respectively) and CUPH group (c-Fos, 21%, *p* < 0.001; c-Jun, 29%, *p* < 0.01, respectively) were significantly decreased. Compared with the control group, MAPK proteins including p-p38, p-ERK, and p-JNK were significantly increased in the DSS group (1.25-fold, *p* < 0.001; 1.76-fold, *p* < 0.001; 1.39-fold, *p* < 0.001, respectively), and compared to the DSS group, the SASP and CUPH groups significantly decreased p-p38 by about 18%, p-ERK by about 39%, and p-JNK by about 17%.

### 3.7. CUP Suppressed NF-*κ*Bp65 and Inflammatory-Related Proteins in DSS-Induced Colon Tissue

The levels of p-I*κ*B*α*, NF-*κ*Bp65, and inflammatory-related proteins including iNOS, Cox-2, TNF-*α*, IL-6, and IL-1*β* were evaluated through Western blotting (Figure 7). Compared with the control group, p-I*κ*B*α* and NF-*κ*Bp65 were significantly increased in the DSS group (1.44-fold, *p* < 0.001; 1.65-fold, *p* < 0.001, respectively), and compared to the DSS group, the SASP group and CUPH group had significantly decreased p-I*κ*B*α* by about 28% and NF-*κ*Bp65 by about 17%. Compared with the control group, iNOS, Cox-2, TNF-*α*, IL-6, and IL-1*β* were significantly increased about 1.30-fold in the DSS group (*p* < 0.01, respectively), whereas compared to the DSS group, the SASP group and the CUPH group were significantly reduced similar to the level of the control group.

### 3.8. CUP Regulated Apoptotic-Related Proteins in DSS-Induced Colon Tissue

The levels of Bax, Bcl-2, caspase-3, and survivin were evaluated through Western blotting (Figure 8). The levels of Bax, Bcl-2, caspase-3, and survivin were evaluated through Western blotting (Figure 8). Compared with the control group, Bax and caspase-3 were significantly increased in the DSS group (1.51-fold, *p* < 0.01; 2.98-fold, *p* < 0.001, respectively), whereas compared to the DSS group, those in the SASP group and the CUPH group were significantly reduced similar to the level of the control group. Also, compared with the control group, antiapoptotic proteins such as Bcl-2 and survivin were significantly decreased in the DSS group (0.38-fold, *p* < 0.01; 0.25-fold, *p* < 0.001, respectively), whereas compared to the DSS group, those in the SASP group and the CUPH group were significantly increased similar to the level of the control group.

## 4. Discussion

Gastrointestinal (GI) diseases, including inflammatory bowel disease (IBD), are diseases that 4–5% of the world's population experience at least once in their lifetime [25], and according to Avraamides's study, 14.6–27.6% of people over the age of 28 years showed a high prevalence [26]. Treatments for inflammatory bowel disease, including ulcerative colitis (UC), can cause various side effects and complications when used for a long time [27]. Therefore, as an alternative to this, new treatments using various natural products are being actively developed [18, 28]. The peel of mature *Citrus unshiu* contains various physiologically active substances such as flavonoids, amino acids, and carotenoids and has been widely used as herbal medicine to treat various diseases [29]. As a result of HPLC analysis using *Citrus unshiu* peel water extract, hesperidin and narirutin, which are flavonoids with anti-inflammatory and antioxidant effects, were detected at 12.210 ± 0.311 and 9.998 ± 0.146 mg/g, respectively. Based on these results, in this study, UC was induced through sodium dextran sulfate (DSS) [30, 31], which is widely used to study the mechanism of UC, and the effect and mechanism of *Citrus unshiu* peel were confirmed.

The reduction in body weight and colon length, typical features of UC, can be corroborated by several cumulative studies of mice exposed to DSS [32–34]. In order to confirm the effect of CUP in the UC model induced by DSS, weight change and colon length during the experimental period were checked. Although the weight change was significantly suppressed in the drug administration group, the decrease in colon length did not appear to be significant, but it showed a tendency to suppress. These results are expected to alleviate UC by suppressing the decrease in body weight and colon length, which are typical features of UC, by CUP to some extent. Myeloperoxidase (MPO), an enzyme mainly present in neutrophils, is an important mediator of several inflammatory responses through the production of specific oxidative species [35]. As a result of measuring the level of MPO in serum in this study, it was confirmed that the level was significantly reduced due to CUP treatment. These results suggest that CUP treatment will suppress the inflammatory response by reducing the activity of MPO, an inflammatory biomarker. As a result of histological analysis through H&E staining of colon tissue, compared with normal colon tissue, loss of colonic muscle fragments and excessive inflammatory cell infiltration were observed in the control group, whereas inflammatory lesions including loss of colonic muscle fragments and inflammatory cell infiltration were reduced in both the SASP group and the CUP-treated groups. The loss of colonic muscle and inflammatory cell infiltration confirmed by H&E analysis of these colon tissues can be confirmed as a result of ulcerative colitis induction in previous studies [33], and the reduction of these symptoms suggests that CUP alleviated UC.

Glutamic oxaloacetic transaminase (GOT) and glutamate pyruvate transaminase (GPT) enzymes are mainly present in hepatocytes, and the enzymes are released into the bloodstream when disease or damage occurs in body tissues and organs such as the liver or heart [36]. Therefore, it can be confirmed by accumulated studies that the increase in GOT and GPT levels is directly related to liver dysfunction and tissue damage [37–39]. Therefore, in this study, it was checked whether liver damage caused by DSS, sulfasalazine, and CUP was observed. As a result of the analysis, treatment with sulfasalazine and CUPH significantly inhibited the increase in GOT and GPT levels. These results suggest that sulfasalazine and CUP not only did not cause liver damage in the UC model but also alleviated the increased GOT and GPT levels due to DSS.

Oxidative stress (OS) results from an imbalance in the antioxidant system, overproduction of reactive oxygen species (ROS), and lipid peroxidation of cell membranes. Overproduced ROS adversely affects biomolecules such as DNA, RNA, proteins, and enzymes [40]. Mitochondria play a significant role in apoptosis initiation, ROS formation, and energy metabolism [41]. When malondialdehyde (MDA) and ROS are accumulated in mitochondria by stimuli such as inflammation, stress, and infection and the activity of antioxidant enzymes is inhibited, the balance of the oxidation-antioxidant system is disrupted, and oxidative stress damage occurs [42]. NADPH oxidase (NOX) is found in the cytoplasm and plasma membrane and plays a key role in generating ROS as a mediator of signaling related to growth, angiogenesis, and apoptosis [43]. Among the NOX subunits, NADPH oxidase-2 (NOX2) produces H_2_O_2_, a metabolite of ROS (here, p47_phox_ and p22_phox_). The interaction is associated with NOX2 activation [44]. In a recent study, inhibition of NOX2, an OS-related protein, improved OS and showed GI protective effects [45]. In addition, a study by Morsy et al. showed that inhibition of MDA and NOX improved colitis [46]. Therefore, in this study, serum ROS and tissue MDA levels were analyzed in the UC model and significant results were obtained from CUP treatment. In addition, the expression of ROS-producing NADPH oxidase-related proteins, NOX2 and p47^phox^, was significantly reduced by CUP treatment. These results suggest that increased OS due to DSS induction was inhibited by CUP treatment, suggesting that UC will be alleviated.

The PI3K/Akt signaling pathway is known to regulate I*κ*B*α* phosphorylation and NF-*κ*Bp65 [47]. These pathways are implicated in multiple cellular processes such as survival, proliferation, differentiation, and apoptosis by directly phosphorylating apoptosis-associated proteins or regulating the activity of transcription factors. Also, Akt is activated as a result of the stimulation of lipopolysaccharide receptors and proinflammatory cytokines [48]. In addition, accumulating evidence shows that the PI3K/Akt signaling pathway acts as a central cell determinant of apoptosis mediated by ROS generation, which is accompanied by activation of the PI3K/Akt signaling pathway [49]. Studies on improving colitis by regulating the PI3K/Akt signaling pathway are actively in progress [31, 50]. Besides, studies such as bladder cancer, gastritis, and Crohn's disease on the regulation of the PI3K/Akt signaling pathway have also been reported [47, 51, 52]. In this study, the expression of PI3K and Akt in the tissues of the UC models was measured, and significant results were confirmed due to CUP treatment. These results suggest that CUP treatment may have improved UC by regulating the PI3K/Akt signaling pathway that causes inflammation, ROS-mediated oxidative damage, and apoptosis.

c-Fos and c-Jun are transcription factors that regulate cellular processes such as cell differentiation, cell proliferation, and apoptosis. These transcription factors are regulated gene expression through responses such as growth factors, stress, cytokines, and stimuli such as bacterial infection. In addition, it is translocated to the nucleus by mitogen-activated protein kinase (MAPK), including p38, ERK, and JNK, to induce the transcription of proinflammatory proteins and play an important role in mediators responsible for the inflammatory response [53]. ERK is related to cell proliferation or differentiation, and p38 and JNK are closely related to stress, apoptosis, and inflammatory response and thus are recognized as key factors regulating inflammation [54]. In addition, the expression of MAPK proteins including c-Fos, c-Jun, p-p38, and JNK was significantly decreased by CP treatment, but in the case of ERK, only CPH showed a significant result. These results suggest that CUP will alleviate UC by inhibiting c-Fos, c-Jun, and MAPK and inhibiting inflammation and stress in the UC model.

NF-*κ*Bp65 binds to I*κ*B*α* in the cytoplasm and exists in an inactive state. When the PI3K/Akt signaling pathway and MAPK are activated, I*κ*B*α* phosphorylation occurs and NF-*κ*Bp65 translocates to the nucleus. After which it transcripts various inflammatory factors [55]. The activated NF-*κ*Bp65 promotes the expression of proinflammatory mediators and proinflammatory cytokines [56]. Therefore, in this study, the expression of p-I*κ*B*α*, NF-*κ*Bp65, inflammatory mediators, and proinflammatory cytokines was analyzed. As a result of the analysis, CUPH treatment showed significant results in the UC model. These results suggest that CUP will alleviate UC by inhibiting inflammatory mediators and proinflammatory cytokines through the inactivation of NF-*κ*Bp65 due to the regulation of the PI3K/Akt signaling pathway.

Intestinal epithelial cells (IECs) are one of the components of the intestinal epithelial barrier. IEC prevents the entry of pathogens and bacterial toxins. Shi's study showed that apoptosis disrupts the intestinal epithelial barrier integrity system and promotes the intestinal inflammatory response [57], and IECs apoptosis was found to be particularly increased in UC patients [58]. In the apoptosis pathway, the ratio of antiapoptotic factor Bcl-2 and proapoptotic factor Bax determines cell growth or apoptosis, and caspase-3, a downstream mediator of Bax, plays a role in inducing apoptosis [59]. Survivin is a small component of antiapoptosis and inhibits apoptosis by degrading caspase-3 [60]. In this study, the expression of proapoptotic proteins such as Bax and caspase-3 was significantly suppressed in colonic tissue by CUP treatment, and the expression of antiapoptotic proteins such as Bcl-2 and survivin was increased. These results suggest that CUP treatment will improve UC by significantly regulating the expression of apoptosis-related proteins in the colon tissues of the UC model.

## 5. Conclusions

Taken together, the improvement effect of CUP on ulcerative colitis was revealed through inflammatory protein and apoptosis by inhibition of PI3K/Akt signaling pathway and MAPK and NF-*κ*Bp65 as shown in Figure 9. Moreover, CUP did not impair liver function and effectively alleviated UC through the PI3K/Akt signaling pathway. These results suggest that CUP containing hesperidin and narirutin, which has excellent anti-inflammatory and antioxidant effects, has potential as a candidate for the development of a UC treatment, and it is judged that it has laid the scientific foundation for future clinical trials. However, in order to clarify the efficacy of CUP for gastrointestinal diseases, additional studies on gastrointestinal diseases including UC using its components hesperidin and narirutin are needed, and an understanding of the precise mechanisms of each is required.

## Figures and Tables

**Figure 1:** Analysis of narirutin and hesperidin in the water extract of *Citrus unshiu* peel. (a) Chemical structure of narirutin; (b) chemical structure of hesperidin; (c) the chromatogram of the extract of CUP. CUP: *Citrus unshiu* peel water extract.

**Figure 2:** *Citrus unshiu* peel improved changes in body weight, colon tissue length, and histological analysis in UC. (a) Change body weight; (b) change in colon length; (c) MPO (myeloperoxidase); (d) histological analysis; (e) histological score. Hematoxylin and eosin (H&E) staining. Blue arrows indicate inflammatory cells infiltration. Magnification ×100 and ×200 (scale bar = 100 *μ*m). Histological analysis was measured using ImageJ program (NIH). Control: control mice, DSS: distilled water administered to ulcerative colitis mice, SASP: sulfasalazine 100 mg/kg body weight administered to ulcerative colitis mice, CUPL: CUP 100 mg/kg body weight administered to ulcerative colitis mice, and CUPH: CUP 200 mg/kg body weight administered to ulcerative colitis mice. Data are mean ± SD (*n* = 8). Significance: ^##^*p* < 0.01 and ^###^*p* < 0.001 vs. control mice, ^*∗*^*p* < 0.05, ^*∗∗*^*p* < 0.01, and ^*∗∗∗*^*p* < 0.001 vs. DSS mice.

**Figure 3:** *Citrus unshiu* peel alleviated the levels of GOT and GPT in UC. (a) GOT (glutamic oxaloacetic transaminase); (b) GPT (glutamate pyruvate transaminase). Control: control mice, DSS: distilled water administered to ulcerative colitis mice, SASP: sulfasalazine 100 mg/kg body weight administered to ulcerative colitis mice, CUPL: CUP 100 mg/kg body weight administered to ulcerative colitis mice, and CUPH: CUP 200 mg/kg body weight administered to ulcerative colitis mice. Data are mean ± SD (*n* = 8). Significance: ^##^*p* < 0.01 and ^###^*p* < 0.001 vs. control mice, ^*∗*^*p* < 0.05, ^*∗∗*^*p* < 0.01, and ^*∗∗∗*^*p* < 0.001 vs. DSS mice.

**Figure 4:** *Citrus unshiu* peel alleviated the levels of oxidative stress biomarkers and NADPH-related proteins. (a) Level of ROS (reactive oxygen species) in serum; (b) level of MDA (malondialdehyde) in tissue; (c) expression of NOX2 (NADPH oxidase 2) and p47^phox^. Control: control mice, DSS: distilled water administered to ulcerative colitis mice, SASP: sulfasalazine 100 mg/kg body weight administered to ulcerative colitis mice, CUPL: CUP 100 mg/kg body weight administered to ulcerative colitis mice, and CUPH: CUP 200 mg/kg body weight administered to ulcerative colitis mice. Data are mean ± SD (*n* = 8). Significance: ^##^*p* < 0.01 and ^###^*p* < 0.001 vs. control mice, ^*∗*^*p* < 0.05, ^*∗∗*^*p* < 0.01, and ^*∗∗∗*^*p* < 0.001 vs. DSS mice.

**Figure 5:** *Citrus unshiu* peel modulated the PI3K/Akt signaling pathway. Control: control mice, DSS: distilled water administered to ulcerative colitis mice, SASP: sulfasalazine 100 mg/kg body weight administered to ulcerative colitis mice, CUPL: CUP 100 mg/kg body weight administered to ulcerative colitis mice, and CUPH: CUP 200 mg/kg body weight administered to ulcerative colitis mice. Data are mean ± SD (*n* = 8). Significance: ^###^*p* < 0.001 vs. control mice, ^*∗∗∗*^*p* < 0.001 vs. DSS mice.

**Figure 6:** *Citrus unshiu* peel inhibited transcription factors such as c-Fos and c-Jun and MAPK. Control: control mice, DSS: distilled water administered to ulcerative colitis mice, SASP: sulfasalazine 100 mg/kg body weight administered to ulcerative colitis mice, CUPL: CUP 100 mg/kg body weight administered to ulcerative colitis mice, and CUPH: CUP 200 mg/kg body weight administered to ulcerative colitis mice. Data are mean ± SD (*n* = 8). Significance: ^###^*p* < 0.001 vs. control mice, ^*∗*^*p* < 0.05, ^*∗∗*^*p* < 0.01, and ^*∗∗∗*^*p* < 0.001 vs. DSS mice.

**Figure 7:** *Citrus unshiu* peel inhibited NF-*κ*Bp65, inflammatory mediators, and proinflammatory cytokines. Control: control mice, DSS: distilled water administered to ulcerative colitis mice, SASP: sulfasalazine 100 mg/kg body weight administered to ulcerative colitis mice, CUPL: CUP 100 mg/kg body weight administered to ulcerative colitis mice, and CUPH: CUP 200 mg/kg body weight administered to ulcerative colitis mice. Data are mean ± SD (*n* = 8). Significance: ^##^*p* < 0.01 and ^###^*p* < 0.001 vs. control mice, ^*∗*^*p* < 0.05, ^*∗∗*^*p* < 0.01, and ^*∗∗∗*^*p* < 0.001 vs. DSS mice.

**Figure 8:** *Citrus unshiu* peel regulated antiapoptotic and proapoptotic proteins. Control: control mice, DSS: distilled water administered to ulcerative colitis mice, SASP: sulfasalazine 100 mg/kg body weight administered to ulcerative colitis mice, CUPL: CUP 100 mg/kg body weight administered to ulcerative colitis mice, and CUPH; CUP 200 mg/kg body weight administered to ulcerative colitis mice. Data are mean ± SD (*n* = 8). Significance: ^#^*p* < 0.05, ^##^*p* < 0.01, and ^###^*p* < 0.001 vs. control mice, ^*∗*^*p* < 0.05, ^*∗∗*^*p* < 0.01, and ^*∗∗∗*^*p* < 0.001 vs. DSS mice.

**Figure 9:** Possible mechanism of *Citrus unshiu* peel in DSS-induced ulcerative colitis. DSS: dextran sulfate sodium; UC: ulcerative colitis; CUP: *Citrus unshiu* peel.

## Data Availability

All data are contained within the article.
